The article "Application of Rapid Rehabilitation Nursing in Thoracic Surgery Nursing" was retracted in 2022. Reason: concerns about the peer review.

# Application of Rapid Rehabilitation Nursing in Thoracic Surgery Nursing

**DOI:** 10.1155/2021/6351170

**Published:** 2021-09-02

**Authors:** Hongliu Liang, Jing Huang, Jijia Tong, Jinyue Wang

**Affiliations:** ^1^Cancer Hospital of China Medical University, Liaoning Province, Shenyang 110042, China; ^2^Liaoning Cancer Hospital and Institute, Liaoning Province, Shenyang 110042, China

## Abstract

To study the application effect of rapid rehabilitation nursing intervention in thoracic surgery nursing, this paper researches controlled trials. First, this paper sets up a control group and a test group. The control group uses traditional nursing methods for thoracic surgical nursing intervention, and the test group adds rapid rehabilitation nursing intervention based on traditional nursing intervention. In addition, the operation and rehabilitation conditions of the control group and the test group are the same. Moreover, this paper records rehabilitation information in real time, performs data processing through statistical methods, and conducts follow-up surveys on the rehabilitation process of patients. In addition, this paper compares nursing effects through data comparison and histogram comparison. From the research results, various parameters of the patient's recovery process and the user satisfaction of the rapid rehabilitation can be seen. Furthermore, nursing is higher than those of the control group, which shows that the rapid rehabilitation nursing method can positively affect the nursing of thoracic surgery.

## 1. Introduction

Surgery is a great trauma to patients in thoracic surgery. Compared with other surgeries, thoracic surgery has the most pain and irritation sources, including surgical incision, destruction of ribs and sternum, rib (sternum) bone spreader damage to chest wall intercostal nerve, cutting of chest wall muscle intercostal muscle, and stimulation and compression of the thoracic drainage tube. The conduction pathways of these noxious stimuli are numerous and complex. Therefore, it brings great pain to postoperative patients. Thoracic surgery is the most painful of all surgical operations. The pain not only brings great pain to the patient but also produces a series of pathophysiological reactions that are not conducive to the patient's postoperative recovery. Wang Tong et al. showed in the study that after thoracic surgery, patients can inhibit breathing due to pain, which induces tachyarrhythmia. Pain is unbearable for patients, and it is also an urgent problem in comfort care [1].

The most common disease in thoracic surgery is lung cancer. According to reports, lung cancer patients account for about 40% of thoracic surgery patients. The second disease is cancer of the esophagus and gastric cardia, and there are relatively few benign diseases of the lung and esophagus. Finally, mediastinal diseases are mainly mediastinal tumors and cysts, of which thymoma is more common.

The incidence of esophageal cancer in our country is relatively high, and about 60% of esophageal cancers in the world occur in China; esophageal cancer deaths account for 23% of all tumor deaths in China. In recent years, the incidence and mortality of esophageal cancer and gastric cardia cancer have shown a slow downward trend in our country. This is inseparable from our country's emphasis on the prevention and control of esophageal cancer and the continuous improvement of residents' nutritional status, living habits, and living environment.

Due to the many tissues and organs of the mediastinum, the source of embryos is complex, and many types of tumors and cysts can occur. Chinese's common primary mediastinal tumors are thymoma, neurogenic tumor, teratoma, various mediastinal cysts, and intrathoracic goiter. Most of the primary mediastinal tumors are benign, and a small part are malignant. Regardless of benign or malignant primary mediastinal tumors, as long as there is no clear distant metastasis and respiratory and circulatory dysfunction, patients should be operated on as soon as possible and strive to remove the tumor [2].

There are many kinds of monitoring and drainage tubes for patients after thoracic surgery, such as ECG monitoring, oxygen inhalation catheter, chest tube, urinary tube, and gastrointestinal drainage tube. In particular, the indwelling of the chest tube and the urinary tube brings a very uncomfortable feeling to the patient. Moreover, the chest tube is also one of the leading causes of postoperative pain in patients [3].

Experts believe that preoperative fear and excessive anxiety can lower patients' pain threshold and make them feel more intense pain during or after surgery and feel less self-conscious about the results of surgery. Patients whose preoperative anxiety level is too low, due to their psychological coping mechanisms of avoidance and denial and lack of due psychological preparation, can easily regard the actual painful experience caused by the operation as a serious blow after undergoing the operation. On the other hand, patients with a moderate level of preoperative anxiety can psychologically have a correct understanding and adequate preparation for the operation and the various problems caused by it. As a result, they can better adapt to the various conditions of the operation and the operation. Moreover, the patient feels well after the operation, and the body recovers more smoothly. However, studies have also shown that the high anxiety response of surgical patients is not limited to the preoperation, nor does it end after the operation, and many patients still have a higher level of anxiety experience after the operation. Moreover, some patients may have a series of pathological psychological reactions after surgery, which affects the prognosis. The common pathological psychological reactions mainly include postoperative consciousness disorder, postoperative psychosis recurrence, and postoperative depression.

## 2. Related Work

Thoracic surgery is traumatic and takes a long time. During the operation, the lung lobes are often squeezed to expand the surgical field of vision. In addition, the free lung and esophagus are often stabbed or irritated to the lung hilum and bronchi, which reflexively causes respiratory secretions to increase. Moreover, postoperative diaphragm injury and chest and stomach dilatation reduce the effective breathing area, which inevitably leads to a decline in respiratory function and respiratory complications [4].

The literature in [5] believed that cricothyrocentesis can improve the ability of patients to expectoration after thoracotomy. The traditional acupressure cricothyroid technique stimulates cough and expectoration, which is more painful. Repeated pressing and stimulation can easily lead to local tissue edema and aggravation of pain, but some patients are not sensitive.

The literature in [6] investigated the discomfort and needs of 31 thoracotomy patients during the perioperative period. The results showed that, under the condition of continuous analgesia, 16% of patients felt severe pain in the incision of the closed thoracic drainage tube 24 hours after the operation. However, when the tube was removed, the pain gradually disappeared. Both the irritation produced by the indwelling catheter after surgery and the pain of peeing after the catheter is withdrawn have been documented in the literature.

The literature in [7] proposed the application of rapid card rehabilitation nursing in thoracic surgery nursing. The purpose is to achieve rapid recovery of patients and shorten the length of hospital stay. The literature in [7] studied the impact of perioperative care for patients with noncardiac surgery on morbidity, mortality, and other outcome indicators and formally proposed the concept of ERAS. Moreover, it proposed that improving multimodal interventions in the context of fast-track surgical planning is the main challenge for medical professionals in their efforts to achieve perioperative pain and risk-free.

With the growing desire for fast recovery, surgical methods have grown more advanced, perioperative care has become less intrusive, and physicians have started to try to minimize patients' postoperative stress reactions. Accelerated rehabilitation surgery has also emerged [8]. However, surgery, as a treatment method, also has elements of intentional injury. Trauma mediated by cytokines, nitric oxide, and free oxygen free radicals can cause psychological and physiological changes in the patient's body and cause additional damage to normal tissues. However, multimodal interventions can counter the stress response of surgical operations and are believed to reduce the adverse effects of surgical injury and accelerate the recovery of patients. At present, the most effective intervention measures are as follows: restore diet as soon as possible, avoid mechanical intestinal preparation, preoperative patient education, reduce complications, avoid hypothermia, and use the least drugs.

Invasive surgery, preventing surgical site infections and venous thromboembolism and ensuring optimal analgesia, is a new minimally invasive rehabilitation treatment model, including three connotations of psychological minimally invasive, functional minimally invasive, and structural minimally invasive. It pays more attention to humanistic care, adheres to the patient as the main body, optimizes implementing many old perioperative treatment measures, and gradually forms a theoretical system with evidence-based medicine. Moreover, based on the immediate interests of patients, it cooperates with multiple departments such as surgery, nursing, and anesthesia and provides safe, accurate, and minimally invasive medical technology while reducing the physical and physiological trauma to patients. In addition, it reduces the incidence of postoperative complications of patients, speeds up recovery, shortens the length of hospitalization, reduces patient hospitalization costs, improves patient satisfaction, conforms to the national medical reform trend, eases doctor-patient conflicts, and increases social benefits [9].

After the patient is admitted to the hospital, it is necessary first to assess the patient's nutritional status and physical condition, as well as actively communicating with the patient and their family members, to determine whether the patient is suitable for the application of the ERAS concept and to assess the expected effects and potential risks that can be achieved by doing so. For patients with malnutrition, cardiovascular disease, or other underlying diseases, multidisciplinary consultation is needed to correct the patient's basic state and determine whether the patient can enter the ERAS group-related pathways [10]. Literature [11] believed that when patients with no malnutrition, heart, brain, lung, kidney, and other organ dysfunction diseases are included in the ERAS management model, they can recover more quickly after surgery. However, the ERAS management model is not recommended for patients with malnutrition, basic organ dysfunction, acute abdomen, and severe abdominal adhesions. The literature [12] also proposed that, during the perioperative period of cesarean section, pregnant women with high-risk factors such as premature rupture of membranes, placenta previa, eclampsia, and placental abruption do not recommend ERAS management. The literature [13] believed that giving nutritional support to severely malnourished patients before surgery can effectively reduce postoperative complications by 50%. At present, most ERAS studies, for the sake of safety and precaution, subconsciously exclude elderly patients with many comorbidities. However, a colorectal surgery study of 188 elderly patients with colon cancer over the age of 70 showed that the incidence of postoperative complications, secondary hospitalization, and operation rates in elderly patients did not increase, which proved that the application of ERAS in the elderly group is also feasible and safe [14]. Other related clinical studies have also shown that ERAS is also safe and effective in emergency surgery for colorectal cancer complicated by intestinal obstruction [15]. Many guidelines have also pointed out that ERAS is to benefit patients the most, with minimal harm, without absolute contraindications, and ERAS should be a concept, not a step-by-step model. Therefore, when applying the ERAS concept, the diagnosis and treatment plan should be individualized according to the patient's condition and physical condition, and the intervention measures should be flexibly adjusted [16].

## 3. Materials and Methods

We select 200 patients from 428 thoracic surgery patients in a hospital from January 2019 to March 2021, of which 55 are lungs and 145 are esophageal surgery. Moreover, there are 150 males and 50 females, and the age range is 31–79 years. The common symptom characteristics of the included cases are as follows: the patient is conscious, the cardiopulmonary function test before the operation is normal, the male smoker has quit smoking for more than 2 weeks, and there is no history of diabetes. Moreover, all cases are anesthetized with double-lumen bronchial intubation, fentanyl + propofol intravenous anesthesia, and penicillin antibiotics are used 1 day before and during the operation. Exclusion criteria are as follows: patients with chronic heart and lung insufficiency, diabetes, severe obesity, severe malnutrition, wound infections, bleeding, thrombotic veins or lymphitis, and varicose veins and patients who cannot tolerate vibration. According to the principle of randomization, they are divided into two groups: on the basis of conventional treatment, the control group (100 cases) used conventional back-patching to assist sputum, and the test group (100 cases) used a vibration sputum machine to assist sputum (Table 1) [17].

The following nursing methods were used to intervene in the test group and the control group [18].

### 3.1. Control Group

The patient takes the side lying or semisitting position, the operator's five fingers are put together, and the metacarpophalangeal joints are flexed at 120–150. After that, the nurse uses the strength of the wrist joint to strike from the bottom of the lung from the outside to the inside and from the bottom to the top at a frequency of 40–50 beats per minute through the front chest or back. The adjacent parts of the spike should overlap, and the strength should be so strong that the sputum can be discharged smoothly and the patient can bear it. While slamming, the nurse instructs the patient to effectively cough and expectorate, take a deep breath, and cough at about 1/3 of the inhalation. This process is repeated several times. If the patient's cough response is weak, the nurse needs to use a finger to slightly press the junction of the lower edge of the cricoid cartilage and the sternum to stimulate the patient to cough at the end of inhalation. Or, the nurse slightly presses the trachea of the suprasternal fossa of the patient and slides laterally at the same time, which can be repeated several times to stimulate the trachea to prompt the patient to cough up deep sputum. When knocking, the nurse knocks the air between the palm of the patient's hand and the patient's chest wall, so that each knock produces a hollow sound but does not make the patient feel pain. The more air the nurse knocks on, the more effective the knock. The nurse turns the patient over to change position every 2 hours. When turning over, the nurses need to pay attention to placing the patient's limbs in a functional position, and two nurses will knock on the patient's back. The number of taps per day is 4 times; each time is 15 min to 20 min [19].

### 3.2. Test Group

The test group adopts the same nursing methods as the control group in terms of basic nursing methods. On this basis, nursing intervention is also carried out through rapid rehabilitation nursing. In addition, some current perioperative nursing routines, such as smoking cessation before surgery, the use of preventive antibiotics, the maintenance of intraoperative body temperature, and the prevention of deep vein thrombosis, were found to be in line with the concept of accelerated rehabilitation surgery during the implementation process.

There is no change to this part that is consistent with the concept of accelerated rehabilitation surgery. However, preoperative education, preoperative medication, preoperative fasting, preoperative bowel preparation, intraoperative fluid control, postoperative analgesia, and early postoperative activities should be changed that are inconsistent with the concept of accelerated rehabilitation surgery. Therefore, we have developed a clinical nursing path for accelerated rehabilitation surgery for patients with single lobectomy. Before implementing the rapid recovery surgery concept and clinical nursing path intervention plan for patients with thoracoscopic single lobectomy, all members of the rapid recovery management team of thoracic surgery need to be trained in relevant theoretical knowledge and pass the assessment. The clinical nursing path of rapid rehabilitation surgery conducts a small-scale preexperiment before use. A department of thoracic surgery was selected for a one-month preexperiment. The purpose of the experiment was to test whether the content in the clinical nursing path table of rapid rehabilitation surgery meets the actual work of our hospital and whether it meets the needs of patients for treatment, nursing, and rehabilitation. During the preexperiment period, 20 rapid rehabilitation clinical nursing paths are completed. According to actual work requirements, the time node is formulated. Patients undergoing thoracoscopic single lobectomy are routinely used for 2 to 3 days according to their condition and need ECG monitoring, and the tube is extubated about 4 to 7 days after the operation. The average length of hospital stays for patients who fully recover and were discharges from the hospital is about 14 days. After the preliminary experiment, the opinions and suggestions of each patient are collected, and the patients and their families are asked to fill in their feelings and rehabilitation needs in the blank space on the last day of the path table. According to the needs of patients and the actual clinical work, the clinical nursing pathway in rapid rehabilitation of surgery is formulated [20].

The department has established a nursing team of a clinical nursing pathway in rapid rehabilitation of surgery with the head nurse and key nurses as the main members and is responsible for the training, guidance, and implementation of the clinical nursing pathway application of rapid rehabilitation surgery in the department. Patients who cannot successfully complete the path are regarded as variant cases, the data is collected regularly, and the cause analysis is done.

Patients in both groups were treated with thoracoscopic single lobectomy. The intervention group used the constructed clinical nursing pathway table in rapid rehabilitation of thoracoscopic single lobectomy to carry out various postoperative nursing, and the control group used the current nursing routine of thoracic surgery [21].

At the same time, a three-level quality control system of “Nursing Department-Major Section-Department” is established to do a solid job of quality inspection. The nursing quality control checklist for clinical nursing pathway in rapid rehabilitation of thoracoscopic single lobectomy is produced. The quality control is carried out from the aspects of “general requirements for on-site inspection and inspection records; inspection of patients and nurses during the implementation process; inspection of patients for health education; implementation of summary inspection of data.” Each responsible nurse checks and scores each medical record of each completed path according to the checklist. In addition, the monthly team leaders will discuss and analyze rectification at the monthly meeting. Quarterly, the nursing department will organize the head nurse of the general surgery and the team leaders to discuss, analyze, and rectify the rectification [22].

## 4. Results

A controlled experiment verifies the effect of rapid rehabilitation nursing in thoracic surgery nursing, the nursing results are counted, and the analysis is carried out as follows.

First, the postoperative recovery time of patients is counted. This article mainly counts the time until the patient can get out of bed and walk on their own after the operation. The results of the control group and the test group are shown in Table 2 and Figure 1.

From the above results, it can be seen that the postoperative recovery time of the test group is 7-9D, while the recovery time of the control group is 9-12D. Therefore, the postoperative recovery effect of the test group was significantly better than that of the control group, and the result was statistically significant.

Next, this paper counts the length of stay in the hospital, and the results are shown in Table 3 and Figure 2.

From the above analysis results, it can be seen that the length of stay in the hospital of the test group patients is basically distributed in 13-15D, while the hospital stay of the control group is distributed in 14-17D. It can be judged that the length of hospital stay in the test group is lower than that in the control group, which also proves that rapid rehabilitation nursing has advantages compared with traditional nursing methods.

Finally, patients' satisfaction is investigated, and the statistical results are shown in Table 4 and Figure 3.

From the above analysis results, it can be seen that the satisfaction of patients in the test group is significantly higher than that of the control group, which proves that rapid rehabilitation nursing has more advantages than traditional nursing methods.

## 5. Conclusion

Before implementing a clinical nursing pathway in rapid rehabilitation of thoracic surgery, this study established a multidisciplinary management team with anesthesiologists, thoracic surgeons, and nurses. The management of pain in the clinical nursing pathway in rapid rehabilitation of thoracic surgery is a joint multidisciplinary cooperative pain management model. Following the path table, nurses in the preoperative ward preached on pain knowledge, and anesthesiologists actively carried out preoperative visits to train patients on pain management related knowledge. During the operation, anesthesiologists carried out multimodal analgesia and actively guided thoracic surgeons to regulate moderate-to-severe postoperative pain management. Thoracic surgeons participate in multimodal analgesia during the operation and scientifically carry out analgesia management under the guidance of anesthesiologists after the operation. Thoracic surgery nurses accurately assess patient pain and carry out nondrug analgesia management. The multidisciplinary cooperative pain management model in the concept of rapid rehabilitation makes full use of the three disciplines resources of anesthesiology, thoracic surgery, and nursing. Moreover, it integrates pain management throughout the perioperative period of patients undergoing thoracoscopic single lobectomy and provides patients with effective postoperative analgesia throughout the entire process. Previous studies have shown that analgesic knowledge education is an important way to improve the effect of postoperative analgesia in patients. It can improve the patient's correct awareness of analgesia, increase the patient's acceptance of postoperative analgesia, improve the patient's demand for postoperative analgesia, and improve the quality of postoperative analgesia. Clinical nursing pathway in rapid rehabilitation of thoracic surgery improves the patient's acceptance of postoperative analgesia and enables them to cooperate with medical staff for treatment actively, thereby shortening the time of getting out of bed, promoting sleep, and being conducive to the recovery of patients' physiological functions.

The patient's recovery is an accumulation process, and the occurrence of complications does not happen suddenly. The design of the clinical nursing path emphasizes the focus of the patient's daily rapid recovery and assists the nurse to observe the patient's condition changes and recovery needs. The clinical nursing path table is hung at the bedside of the patient. It is also a mode of education for the patient and supervises the patient to complete the daily focus of their rehabilitation path in a planned and purposeful manner. Effective implementation of various nursing measures is the key to reducing postoperative complications. The treatment of postoperative complications is the main reason for delayed discharge of patients and increased length of stay in hospital.

In patients undergoing thoracoscopic single lobectomy, the application of clinical nursing pathway in rapid rehabilitation of thoracic surgery strengthens respiratory function exercises and postoperative activity guidance at each time period, relieves postoperative pain levels, enhances patients' awareness of participating in treatments, enables patients to know the surgical treatment and nursing process, eliminates patients' doubts, and improves their compliance. The clinical nursing pathway in rapid rehabilitation of thoracic surgery clearly lists the daily treatment, nursing, and education that patients need to receive. Therefore, nurses reduce the possibility of repeated missions, save time, and improve work efficiency. Moreover, nurses can free up more time to communicate with patients and provide guidance and assistance on problems that patients urgently need to solve, which improves the effectiveness of patients' treatment. In addition, the combination of rapid rehabilitation surgery concept and clinical nursing path is an incentive for patients. The path table is suitable for most patients undergoing thoracoscopic single lobectomy. The corresponding plan is completed every day. As a result, the patient is confident in the recovery and avoids the psychological dependence of the patient after the operation. A number of studies have shown that the recovery effect of patients is better by actively performing exercises and passively receiving instructions. These have improved our traditional mode of communicating with patients and improved patients' overall satisfaction with our nursing services.

## Figures and Tables

**Figure 1:** Statistical diagram of postoperative recovery time.

**Figure 2:** Statistical diagram of the length of stay in the hospital.

**Figure 3:** Statistical diagram of the satisfaction of patients.

**Table 1:** Comparison of clinical data (*n* = 100).

Index	Men and women	Age	Esophageal cancer	Lung cancer	Have a history of smoking
Control group	74/26	57.4	71	29	64
Test group	76/26	58.2	74	26	61
*χ*2/*t*	1.4328	0.4101	0.1524	0.1832	0.1542
*P*	0.2314	0.6841	0.1578	0.1754	0.7254

**Table 2:** Statistical table of postoperative recovery time.

No.	Test group	Control group	No.	Test group	Control group	No.	Test group	Control group
1	7.0	9.6	35	8.8	11.4	68	7.6	11.9
2	7.2	9.2	36	7.6	11.8	69	8.8	11.3
3	8.6	9.9	37	8.0	11.7	70	7.9	11.0
4	8.4	9.8	38	8.9	10.0	71	7.3	11.8
5	8.1	11.9	39	8.9	9.5	72	7.6	11.6
6	7.0	9.6	40	8.4	10.0	73	7.5	10.0
7	7.1	11.3	41	8.6	10.4	74	8.0	11.0
8	9.0	9.7	42	7.2	11.5	75	7.8	9.2
9	8.6	10.0	43	8.6	11.5	76	7.2	9.5
10	8.9	9.7	44	7.5	9.1	77	8.8	11.9
11	7.7	9.7	45	8.8	11.4	78	7.9	10.7
12	8.2	11.9	46	8.7	10.2	79	8.2	10.3
13	7.3	9.5	47	7.8	11.3	80	7.6	11.5
14	7.3	9.8	48	8.9	10.7	81	7.8	9.9
15	8.6	10.5	49	8.8	10.0	82	7.2	9.8
16	7.4	9.4	50	7.4	11.5	83	7.0	11.9
17	7.4	10.9	51	7.7	11.8	84	7.4	11.8
18	7.9	9.7	52	7.7	11.8	85	7.6	11.6
19	8.1	9.9	53	8.5	9.2	86	7.4	10.4
20	7.4	9.1	54	8.7	10.0	87	7.8	11.4
21	8.9	9.1	55	7.1	10.1	88	7.5	9.1
22	8.8	9.1	56	8.8	11.4	89	7.1	9.3
23	7.7	11.1	57	8.3	11.3	90	8.5	11.3
24	7.7	9.6	58	8.7	10.4	91	7.2	9.4
25	7.8	10.5	59	7.7	11.2	92	8.7	11.0
26	8.3	10.9	60	7.5	9.3	93	9.0	10.6
27	8.9	11.7	61	7.2	10.6	94	7.3	11.9
28	9.0	9.5	62	8.7	11.3	95	8.8	11.5
29	7.9	9.2	63	8.5	10.2	96	7.9	10.1
30	8.6	11.5	64	8.8	11.8	97	7.1	11.6
31	7.3	10.2	65	8.7	9.4	98	8.7	9.0
32	8.9	11.1	66	8.4	11.3	99	7.5	11.3
33	8.2	9.5	67	8.4	9.9	100	9.0	10.4
34	8.2	9.1						

**Table 3:** Statistical table of the length of stay in the hospital.

No.	Test group	Control group	No.	Test group	Control group	No.	Test group	Control group
1	13.2	16.6	35	14.3	15.0	68	14.6	15.4
2	14.9	14.4	36	14.1	14.9	69	14.2	17.9
3	14.2	14.0	37	13.2	14.2	70	13.5	17.3
4	14.9	14.0	38	14.4	16.7	71	14.6	16.7
5	13.0	16.3	39	13.7	16.2	72	14.4	15.7
6	14.6	15.8	40	14.1	15.9	73	14.1	16.4
7	14.3	15.4	41	14.2	17.7	74	14.8	17.0
8	13.8	15.8	42	13.1	17.6	75	14.5	14.7
9	13.3	16.3	43	13.0	17.5	76	14.4	16.0
10	14.8	15.2	44	14.3	17.3	77	14.6	17.7
11	14.7	15.5	45	14.9	15.6	78	13.2	15.5
12	14.9	14.8	46	14.4	14.3	79	13.8	15.0
13	14.3	16.3	47	13.3	16.5	80	14.1	15.3
14	14.0	15.7	48	14.5	16.1	81	13.8	15.1
15	14.0	17.1	49	14.8	16.5	82	13.8	14.4
16	14.9	15.8	50	13.4	16.2	83	14.6	16.2
17	14.2	14.4	51	13.2	17.8	84	13.8	16.2
18	14.4	16.6	52	13.4	16.5	85	14.2	15.2
19	13.5	17.8	53	14.6	17.6	86	14.7	15.0
20	13.3	16.3	54	14.5	14.4	87	14.7	17.4
21	14.5	16.7	55	13.7	15.1	88	14.1	17.9
22	13.1	15.4	56	13.3	17.4	89	13.3	14.7
23	13.0	14.4	57	13.7	15.7	90	14.9	14.4
24	13.9	14.9	58	14.6	14.5	91	14.4	15.0
25	14.7	15.5	59	13.8	16.3	92	13.8	14.2
26	14.9	16.5	60	14.4	17.9	93	13.2	14.8
27	14.3	17.3	61	13.3	17.0	94	13.1	16.7
28	13.4	15.3	62	13.6	17.8	95	13.2	15.0
29	14.5	15.5	63	13.9	14.4	96	14.8	14.9
30	13.8	16.5	64	13.5	15.1	97	14.2	18.0
31	14.8	16.8	65	13.3	15.4	98	13.6	16.1
32	13.3	17.3	66	15.0	14.7	99	13.7	17.5
33	15.0	17.4	67	14.5	14.1	100	14.3	16.8
34	13.7	17.9						

**Table 4:** Statistical table of the satisfaction of patients.

No.	Test group	Control group	No.	Test group	Control group	No.	Test group	Control group
1	80	89	35	89	69	68	95	83
2	92	80	36	84	82	69	84	60
3	88	82	37	81	59	70	86	65
4	81	70	38	94	87	71	86	87
5	89	82	39	84	59	72	92	88
6	80	73	40	91	69	73	94	69
7	95	84	41	88	76	74	86	68
8	80	80	42	87	81	75	85	85
9	79	60	43	91	82	76	91	87
10	85	70	44	88	76	77	90	91
11	80	91	45	89	60	78	88	72
12	97	66	46	89	79	79	92	65
13	80	65	47	88	63	80	81	62
14	83	89	48	91	69	81	88	86
15	90	74	49	80	69	82	79	77
16	84	85	50	93	64	83	80	87
17	81	75	51	79	87	84	83	60
18	94	91	52	84	60	85	91	82
19	85	87	53	80	86	86	84	67
20	81	78	54	87	82	87	92	90
21	93	74	55	80	63	88	87	72
22	96	79	56	85	63	89	79	64
23	89	75	57	86	82	90	78	72
24	88	76	58	88	87	91	95	61
25	85	68	59	90	76	92	84	63
26	93	85	60	81	68	93	96	91
27	78	77	61	84	65	94	93	81
28	85	83	62	82	74	95	87	69
29	89	91	63	87	77	96	87	74
30	83	89	64	83	58	97	84	80
31	79	78	65	86	64	98	95	60
32	95	73	66	94	84	99	92	60
33	88	82	67	82	65	100	90	59
34	81	60						

## Data Availability

The data used to support the findings of this study are included within the article.
